RETRACTED

# Relationship between Self-Esteem, Interpersonal Trust, and Social Anxiety of College Students

**DOI:** 10.1155/2022/8088754

**Published:** 2022-07-25

**Authors:** Xiahong He

**Affiliations:** Hangzhou Vocational & Technical College, Hangzhou 310018, China

## Abstract

This study attempts to disclose the relationship between self-esteem, interpersonal trust, and social anxiety of college students and provide an empirical reference for enhancing their self-esteem, cultivating their interpersonal trust, and reducing their social anxiety. Specifically, 673 college students were randomly sampled and measured against the self-esteem scale (SES), interpersonal trust scale (TS), and interaction anxiousness scale (IAS). The results show that self-esteem does not vary significantly with genders and origins; social anxiety does not vary significantly with origins but differs significantly between genders; the social anxiety of males is much lower than that of females; interpersonal trust differs significantly between genders and between origins. Self-esteem is significantly correlated with interpersonal trust (*r* = 0.22, *p* < 0.01). Social anxiety has a significant negative correlation with self-esteem (*r* = −0.17, *p* < 0.01) and with social anxiety (*r* = −0.26, *p* < 0.01). Interpersonal trust partly mediates the relationship between self-esteem and social anxiety. These findings provide a theoretical basis for enhancing and improving mental health education of college students.

## 1. Introduction

The college students, who are under the transition from campus life to social life, face various complex social relations and intense competitions. During the transition, the negative emotion of social anxiety often results in retreat, depression, and indifference among the college students. Many studies have attributed anxiety and other emotional problems to interpersonal trust. Meanwhile, self-esteem can be regarded as a regulation mechanism for individuals to face new things. It is the individual experience and understanding of the incidents in his/her living environment. The improvement of self-esteem enables an individual to better perceive the acceptance by others and have a positive emotional experience. In addition, interpersonal trust is the basis for building a good interpersonal relationship.

Many scholars have studied the relationship between college students' social anxiety and self-esteem. However, there is not yet a comprehensive discussion about the psychological mechanism of college students' social anxiety from the perspectives of self-esteem, interpersonal trust, and social anxiety.

Social anxiety refers to the tension and fear of interpersonal situation. Baldwin and Main [1] believed that “fear of judgment” is behind social anxiety, where people worry about what others think of them, especially negative ones. Guo [2] thought that self-evaluation and social skills are the key factors affecting social anxiety. According to epidemiological studies, anxiety grows and differentiates obviously from the normal development in childhood to the socializing in adolescence. Upon entering the adolescence stage, people face changes in two important psychological features. One of them is the strong fear of society, due to the low evaluation of social status. Some researchers have discovered the prevalence of social anxiety among college students [3]. It is one of the most common emotional problems in college, exerting negative effects on many aspects, namely, academic development, career, and interpersonal communication. Abundant evidence has shown that college students' social anxiety comes from various reasons, including the influence of external environment and the subjective feelings of individuals [4–8].

RETRACTED

Rotter defined trust as an expectancy held by an individual or group that the word, promise, and verbal or written statement of another person or group can be relied upon [9]. Wrightsman [10] pointed out that trust is a belief held by individuals that forms part of their personal characteristics. This belief holds that ordinary people are sincere, kind, and trustworthy. Interpersonal trust is a major cause of emotional problems like social anxiety. Domestic and foreign researchers have also verified the high correlation between interpersonal trust and social anxiety. For example, some scholars found that interpersonal trust directly regulates the social anxiety of college students. The relevant studies suggest that social anxiety is greatly affected by the interpersonal trust of individuals in interpersonal communication [11–13].

As an important component of the ego-system of an individual, self-esteem is the positive orientation of an individual towards the evaluation and judgment of self-value through social comparison. The level of self-esteem directly bears on the psychological health and shapes the personality of individuals. For a long time, self-esteem has widely concerned psychologists as a core issue in psychology, sociology, and anthropology. Robins et al. examined the relationship between self-esteem and the Big Five traits and discovered that individuals with a high self-esteem tend to be emotionally stable, highly extravert, and very cautious. Mark R. Leary et al. held that self-esteem helps to monitor interpersonal relationships. A low self-esteem will weaken the individual ability to adapt to the communication environment, easily cause sensitivity to interpersonal rejections, and thus increase the level of social anxiety. Thus, the level of self-esteem is significantly correlated with social anxiety [14–17].

RETRACTED

How to help college students better cope with social confusion in daily life and maintain a good mental health has piqued the interest of all those caring about education and the growth of college students. The previous studies on social anxiety mainly focus on defining concepts, designing questionnaire, setting up evaluation standards, and summing up the features and causes of individual development of social anxiety. There is little report on the relationship between social anxiety, individual self-esteem, and interpersonal interaction. This paper explores the relationship between self-esteem, interpersonal trust, and social anxiety, aiming at providing an empirical reference for enhancing their self-esteem, cultivating their interpersonal trust, and reducing their social anxiety [18–20].

## 2. Methodology

### 2.1. Objects

Stratified random sampling was performed to select undergraduates and junior college students from all four grades in three colleges: Hangzhou Vocational & Technical College, Zhejiang University, and Hebei University of Economics and Business. A total of 700 questionnaires were issued. 673 valid responses were collected, putting the effective rate at 93.5%.

### 2.2. Instruments

#### 2.2.1. Self-Esteem Scale (SES)

Rosenberg's SES was modified by Shen and Cai [14], providing a self-reporting tool of overall self-esteem of individuals. The ten items need to be rated against Likert's 4-point scale. The full mark is 10–40 points. The higher the score, the greater the self-esteem. The Cronbach's alpha of the scale was 0.88. The correlation coefficient remeasured after one week was 0.82.

#### 2.2.2. Interaction Anxiousness Scale (IAS)

The IAS is a self-reporting tool of individual subjective experience of social anxiety. The fifteen items need to be rated against Likert's 5-point scale. The full mark is 15–75 points. The higher the score, the greater the subjectively perceived social anxiety. Among them, items 3, 6, 10, and 15 are reverse scored. The Cronbach's alpha of the scale was 0.87.

#### 2.2.3. Interpersonal Trust Scale (TS)

The TS is a self-reporting tool for those with close relationships to measure their interpersonal trust. The eighteen items need to be rated against Likert's 7-point scale. The full mark is 18–126 points. The higher the score, the greater the trust in interpersonal interaction. The Cronbach's alpha of the scale was 0.81; the predictability a was 0.82; the validity was 0.80.

RETRACTED

## 3. Results

### 3.1. Basic Descriptive Analysis

The 673 effective respondents are aged between 17 and 23. The average age stands at 19.9. In terms of gender, there are 362 females and 311 males. In terms of specialty distribution, 368 respondents major in science and 305 in liberal arts. In terms of origin, 317 respondents come from cities and towns and 356 come from the rural area. When it comes to the number of children in their families, 321 respondents are the only child and 352 have at least one brother or sister. Finally, in terms of grade distribution, quite many respondents are in grade 1; the other respondents are uniformly distributed across grade 2, grade 3, and grade 4. The overall distribution of the respondents is shown in Figure 1.

### 3.2. Analysis on the Level of Each Parameter

As shown in Table 1, the self-esteem of the college students does not vary greatly with genders and origins. There is no significant difference between students of different origins in terms of social anxiety.

The students of different genders and origins differ significantly in interpersonal trust. The interpersonal trust of females is much lower than that of males: females are more unlikely to trust others than males during interpersonal communication. The students from cities and towns have a higher interpersonal trust than those from the rural area: urban students are more likely to trust others than rural students. In addition, the students of different genders vary significantly in social anxiety: males have a much lower social anxiety than females.

### 3.3. Correlation Analysis

As shown in Table 2, there is a significant positive correlation between college students' self-esteem and interpersonal trust (*p* < 0.01): the higher the self-esteem, the greater the interpersonal trust. There is a significant negative correlation between college students' self-esteem and social anxiety (*p* < 0.01): the higher the self-esteem, the weaker the social anxiety. There is a significant negative correlation between college students' interpersonal trust and social anxiety (*p* < 0.01): the higher the interpersonal trust, the lower the social anxiety.

### 3.4. Mediating Effect Analysis

This study discusses the mediating effect of interpersonal trust on the relationship between college students' self-esteem and social anxiety. The mediating effect among self-esteem, interpersonal trust, and social anxiety is analyzed with SPSS Macro (Preacher, 2007). Referring to the demonstration of mediating effect testing by Wen and Ye [21], self-esteem, interpersonal trust, and social anxiety meet the basic conditions for mediating effect analysis. Taking self-esteem as an explanatory variable, interpersonal trust was subjected to a regression analysis. The regression equation was significant (*F* = 33.76, *p* < 0.01), and the standard regression coefficient was 0.22 (*t* = 5.81, *p* < 0.01).  Table 3 lists the analysis results.

RETRACTED

As shown in Table 3, when social anxiety was adopted as an explanatory variable for stratified regression analysis, the inclusion of interpersonal trust weakens the prediction effect of self-esteem on social anxiety. Further, the Sobel test was carried out, revealing the partial mediating effect of interpersonal trust between self-esteem and social anxiety (*z* = 4.22, *p* < 0.01). Then, the mediating effect was fitted by Amos.  Figure 2 shows the mediating effect of interpersonal trust on the relationship between self-esteem and social anxiety. It can be seen that the model achieves a high goodness of fit.  Table 4 lists the fitness indices.

## 4. Discussion

This study shows that, in the process of social interaction, the interpersonal trust of females is lower than that of males. A possible reason is that females have a smaller interpersonal communication range than males and females find it hard to quickly switch to a new relationship, not to mention fully trusting others, due to their high awareness of self-protection and high sentimentality. That is why females generally lag males in interpersonal trust.

In terms of origin, the students from the rural area have significantly lower interpersonal trust than those from cities and towns. This is because the education state of students is closely associated with the growth environment of their origins. Living in a more complex environment, urban students know and understand the interpersonal relationship earlier than their rural counterparts. In addition, rural people often help each other, while urban people keep a distant relationship from each other, which limits the mutual effect between them. In the rural area, the interpersonal communication is largely as frequent as that in the traditional society. Thus, an individual in the rural area is greatly affected by those in his/her surroundings.

In addition, males have a much weaker social anxiety than females. This finding is basically consistent with the roles of the two genders in real life. It can be confirmed that a gender difference exists in the anxiety of college students and females are much more anxious than males.

### 4.1. Relationship between Self-Esteem and Interpersonal Trust

According to the regression analysis with self-esteem as the explanatory variable and interpersonal trust as the explained variable, the regression coefficient of self-esteem relative to interpersonal trust and any of its dimensions reaches the significant level. Self-esteem has an obvious prediction effect of interpersonal trust: a person with a high self-esteem must have a high interpersonal trust.

RETRACTED

Self-esteem can be regarded as a regulation mechanism for individuals facing new things. When the self-esteem increases, an individual would better perceive the acceptance by others and experience positive emotions. Meanwhile, interpersonal trust is the basis for building a good interpersonal relationship. Hence, the self-esteem level of an individual sets the tone for his/her interpersonal trust.

Self-esteem reflects an individual's self-worth and self-acceptance. A high self-esteem is often accompanied by a high self-worth and a high self-acceptance. In the face of new things or people, a high-self-esteem individual would feel his/her value and the love from others through the interaction. Besides, such an individual is very likely to explore the surrounding world, provided that the interaction object is safe. In this way, the individual would trust more in the object, which facilitates the smooth progress of interpersonal communication.

### 4.2. Relationship between Self-Esteem and Social Anxiety

Our study proves that college students' self-esteem has a significant negative correlation with social anxiety. A high social anxiety is closely associated with a low self-esteem. There are two possible reasons:

On the one hand, college students have not developed a perfect internal evaluation system of self-value. Their self-esteem mainly depends on others' attitude. Moreover, college students wish to improve their self-value by winning the recognition from others, especially authoritative people, through socializing. Thus, they attach great importance to the evaluation of others and often worry whether they can be accepted and recognized. This psychology is manifested as social anxiety.

On the other hand, social anxiety is generally anticipatory. In the beginning, this negative emotion takes the form of nervousness, upset, and fear, which are signs of inferior mentalities (e.g., self-denial, lack of security, self-hatred, and self-loathing) in social activities. With a high social anxiety, an individual deeply worries about his/her performance in interpersonal communication and fears that his/her poor performance may invite negative evaluation from others.

Experiments on self-esteem and social anxiety show a significant negative correlation between the two parameters. This agrees with the previous research results.

### 4.3. Influence of Interpersonal Trust on Social Anxiety

This study also examines the relationship between interpersonal trust and social anxiety. It was found that the higher the interpersonal trust, the lower the social anxiety; the lower the interpersonal trust, the higher the social anxiety. For college students, interpersonal trust, or any of its dimensions, has a significant negative correlation with social anxiety. For a considerable number of college students, their social anxiety stems from the distrust of others and the poor ability to live or adapt to the environment.

RETRACTED

Interpersonal trust will directly affect college students' trust in others' behavior, commitment or speech reliability, and affect their emotional state in social communication. With a low interpersonal trust, a college student may hold a highly negative view of the interpersonal communication process and generate an excessive self-defense mentality (e.g., suspicion of and sensitivity to others). Then, many negative emotions would emerge, giving birth to anxiety over communication.

### 4.4. Mediating Effect of Interpersonal Trust between Self-Esteem and Social Anxiety

The regression analysis shows that interpersonal trust partly mediates the relationship between self-esteem and social anxiety. But the mediating effect and mediating variable are largely statistical concepts. The role of the mediating variable is to allow self-esteem to affect social anxiety via interpersonal trust.

Specifically, a high-self-esteem individual has a high self-value and a high self-acceptance. He/she can better perceive the acceptance by others and thus experience positive emotions. Facing new things or people, such an individual would feel his/her value and the love from others through the interaction and willingly explore the surrounding world, provided that the interaction object is safe. In this way, the individual would trust more in the object, which facilitates the smooth progress of interpersonal communication. The smoothness of interpersonal communication, in turn, improves the emotional state of individuals in social interaction and reduces their social anxiety.

## Figures and Tables

**Figure 1:** Distribution of respondents.

**Figure 2:** Mediating effect of interpersonal trust on the relationship between self-esteem and social anxiety.

**Table 1:** Scores of self-esteem, interpersonal trust, and social anxiety (*M* ± SD).

	Male (*n* = 311)	Female (*n* = 362)	*t*-value	Urban area	Rural area	*t*-value
Self-esteem	23.64 ± 2.66	23.60 ± 2.47	0.19	23.59 ± 2.69	23.65 ± 2.43	−0.28
Interpersonal trust	78.65 ± 12.38	75.59 ± 11.11	3.37^∗∗^	78.20 ± 12.51	75.94 ± 11.05	2.48^∗^
Social anxiety	37.05 ± 6.26	38.13 ± 6.29	−2.23^∗^	37.14 ± 6.51	38.06 ± 6.08	−1.88

Standard errors are in parentheses; ^∗^*p* < 0.10, ^∗∗^*p* < 0.05, and ^∗∗∗^*p* < 0.01. *M* and SD are short for mean and standard deviation, respectively.

RETRACTED

**Table 2:** Pearson's correlation coefficients between self-esteem, interpersonal trust, and social anxiety.

	Self-esteem	Interpersonal trust	Social anxiety
Self-esteem	—	0.22^∗∗^	−0.17^∗∗^
Interpersonal trust		—	−0.26^∗∗^

Standard errors are in parentheses; ^∗^*p* < 0.10, ^∗∗^*p* < 0.05, and ^∗∗∗^*p* < 0.01.

**Table 3:** Mediating effect of interpersonal trust on the relationship between self-esteem and social anxiety.

Category	Explanatory variable	*R* ^2^	*F*-score variation	Standard regression coefficient	*t*-value
Step 1	Self-esteem	0.03	19.88	−0.17	−4.46^∗∗^
Step 2	Self-esteem	0.06	22.03	−0.12	−3.14^∗∗^
	Interpersonal trust			0.23	4.85^∗∗^

Standard errors are in parentheses; ^∗^*p* < 0.10, ^∗∗^*p* < 0.05, and ^∗∗∗^*p* < 0.01.

**Table 4:** Fitness indices for the mediating effect of interpersonal trust on the relationship between self-esteem and social anxiety.

*χ* ^2^	df	*χ* ^2^/df	GFI	AGFI	NFI	RFI	IFI	TLI	CFI	RMSEA
88.45	3	29.48	0.99	0.98	0.98	0.96	0.99	0.98	0.99	0.03

*χ* ^2^, df, GFI, AGFI, NFI, RFI, IFI, TLI, CFI, and RMSEA are short for chi square, degree of freedom, goodness of fit index, adjusted goodness of fit index, normal fit index, reproductive fitness index, incremental fit index, Tucker Lewis index, comparative fit index, and root mean square error of approximation, respectively.

## Data Availability

The data used to support the findings of this study are available from the corresponding author upon request.
